The article "Integration of 5G and Block-Chain Technologies in Smart Telemedicine Using IoT" was published in 2021. Journal: J Healthc Eng.

# Integration of 5G and Block-Chain Technologies in Smart Telemedicine Using IoT

**DOI:** 10.1155/2021/8814364

**Published:** 2021-03-22

**Authors:** Kashif Hameed, Imran Sarwar Bajwa, Nadeem Sarwar, Waheed Anwar, Zaigham Mushtaq, Tayyaba Rashid

**Affiliations:** ^1^Department of Computer Science, The Islamia University of Bahawalpur, Bahawalpur 63100, Pakistan; ^2^Department of Computer Science, Bahria University, Lahore, Pakistan

## Abstract

The Internet of Health Thing (IoHT) has various applications in healthcare. Modern IoHTintegrates health-related things like sensors and remotely observed medical devices for the assessment and managment of a patient's record to provide smarter and efficient health diagnostics to the patient. In this paper, we proposed an IoT with a cloud-based clinical decision support system for prediction and observation of disease with its severity level with the integration of 5G services and block-chain technologies. A block-chain is a system for storing and sharing information that is secure because of its transparency. Block-chain has many applications in healthcare and can improve mobile health applications, monitoring devices, sharing and storing of the electronic media records, clinical trial data, and insurance information storage. The proposed framework will collect the data of patients through medical devices that will be attached to the patient, and these data will be stored in a cloud server with relevant medical records. Deployment of Block-chain and 5G technology allows for sending patient data securely at a fast transmission rate with efficient response time. Furthermore, a Neural Network (NN) classifier is used for the prediction of diseases and their severity level. The proposed model is validated by employing different classifiers. The performance of different classifiers is measured by comparing the values to select the classifier that is the best for the dataset. The NN classifier attains an accuracy of 98.98. Furthermore, the NN is trained for the dataset so that it can predict the result of the dataset class that is not labeled. The trained Neural Network predicts and intelligently shows the results with more accuracy than other classifiers.

## 1. Introduction

Telemedicine is a modern technology, and it uses telecommunication that assists a doctor in visiting their patients virtually rather by a live video, an image captured or via email and, receiving patient's information regarding patient's disease [1]. Telemedicine is a means to share resources immediately with any hospital or any doctor in the world. Typically telemedicine works in two ways:

1. Real-time or video
2. Store and forward

In the video method, the patient connects to a specialist on a video call, and the specialist examines the patient's life and suggests treatment. In the store and forward method, the information about the disease of the patient is stored and forwarded to specialists. The minimum time response in the store and forward method is 24–48 hours. In the video method, the response time is zero. But……..!

The article "Integration of 5G and Block-Chain Technologies in Smart Telemedicine Using IoT" was published in 2021. Journal: J Healthc Eng.

In the video method, high-quality cameras are required on the patient and specialist side. For enabling communication between the patient and specialist, the Internet connection must be strong. In developing countries, very expensive, high-quality cameras are not affordable in rural areas. In rural areas, Internet connections are of low quality. So, the video call method for telemedicine is expensive and not practical. Another method is the store and forward method; in this method, the patient stores data about his or her disease and forwards it to the specialist through an expert system by using IoT. The patient visits the health center; the person that runs the health center examines the patient and sends a report to the expert system; the expert system forwards the report to the specialist; the specialist receives the report of the patient and suggests the appropriate treatment through the expert system.  Figure 1 shows the typical store and forward method for telemedicine.

Telemedicine can become more effective by overcoming the critical factors/problems that affect efficiency. The main two factors are

- Time
- Distance

A health center or dispensary that is based on IoT can be at a distance of 15–25 km. For proper treatment, a patient must visit the health center 2–4 times, that is, it takes 3–5 days. The patient that has serious disease needs immediate treatment; otherwise, the patient's health would be dangerously affected. For gaining effective results from telemedicine, the following factors should be considered:

  Hospital: 1–2 days
  Health center: 2–3 days

By minimizing the critical factors of the telemedicine expert system, patients can get immediate treatment. On the expert side, a CDSS system can be installed, which would help in saving time because in the CDSS, the information on the treatment of diseases are stored. When the symptoms of the disease are keyed in, the CDSS matches the information provided with stored information and suggests the treatment within 3–4 minutes. With the enhancement of technology, new viruses and diseases are analyzed and information about diseases is stored in the CDSS. In case a disease appears about which the CDSS has no information, symptoms of the disease are stored and forwarded to a specialist. Treatment of 80% of diseases can be availed through the CDSS. The CDSS helps in minimizing the time factor on the hospital side. The CDSS time is minimized from 1–2 days to 20–30 minutes, and effective response of telemedicine is provided by using IoT.

The article "Integration of 5G and Block-Chain Technologies in Smart Telemedicine Using IoT" was published in 2021. Journal: J Healthc Eng.

To minimize the time and distance factors typically faced ata health center side can be overcomed by using a technology that takes less time such as 5G is faster data transmission medium and can support remote monitoring of smart devices in an efficient manner. The 5G initiative will improve all the hospital processes and of course break the main barrier of Internet bandwidth, creating a truly “Smart hospital.” Normally, visiting the health center 2–3 times will take 2–3 days and a fair amount of distance is also to be covered to visit the health center. So, a mobile application needs to be established. By using a mobile application, one can enter the symptoms of the disease and forward the data to the CDSS or a specialist by using services of 5G, and it will transmit data fast and the patient can get treatment without delay. Different body parameters (blood pressure, the oxygen concentration in blood, pulse rate, body temperature) are calculated and forwarded to the CDSS system. Through mobile application and IoT, and with the integration of block-chain and 5G technologies, time is minimized and data are forwarded within 10 minutes without time-wasting; and through block-chain technologies, data remain secure, even across distances. Block-chain can allow for complete cryptography for the record-keeping of a patient. Block-chain also allows medical records to be stored in secured, fragmented systems that can contain a large amount of data and information, enabling providers to store a more complete patient history and securely encrypt medical data.

By overcoming the critical factors (time, distance), the treatment that would be accessible in 5–6 days can now be availed in 30–40 minutes. Telemedicine effectively improves health by using IoT-based applications, that is, the integration of block-chain with 5G technologies. Now telemedicine can enhance the quality and efficiency of the healthcare system.

 In the propose system's design, it's the consideration that e-Health will improve patient's health monitoring and also provides security in healthcare data management by the use of blockchain technology. The potential of block-chain in healthcare is to overcome the challenges related to data security, privacy, sharing, and storage. Furthermore, block-chain can ensure that medical data are secured in the healthcare system with the utmost transparency.

### 1.1. Contribution of the Paper

In this way, we proposed the cloud-based clinical decision support system using IoT for the prediction and suggested the treatment with its level of severity by implementing the integration of block-chain and 5G technologies. In this proposed system, the patient's data is collected using sensors and data is stored in cloud platform along the patient's medical record from UCI repository by using blockchain technology in which data is stored in blocks.Here, a set of building blocks of a large distributed medical data are formed and resuls of diagnostics are forwarded to the patient by using 5G services. Furthermore, we employ the Neural Network (NN) classifier for the prediction of disease and its level of severity. A different method of the different classifiers is used to train the data and compare the efficiency and accuracy with the NN classifier. Different classifiers are employed to compare the performance of the proposed model. Overall, the contribution of the paper is summarized as follows:

- Present an IoT with the cloud-based framework for the CDSS
- Gather the related medical record of the patient from the UCI repository and also collect the data of different body parameters from Sensors
- Implement the block-chain technologies in storage, which helps to have privacy
- Forward the patient data to healthcare providers by using 5G services
- Employ the NN classifier for identification of the disease
- Compare performance by different classifier values
- Validate the performance of the model by measuring through the different classifiers

The article "Integration of 5G and Block-Chain Technologies in Smart Telemedicine Using IoT" was published in 2021. Journal: J Healthc Eng.

### 1.2. Organization of the Paper

The remaining portion of the paper is arranged as follows: Section 2 surveys the recent IoT-based healthcare application by using different techniques for IoT healthcare.  Section 3 explains the proposed work in a detailed manner with implementation details. Designing of the Neural Network and prediction system is shown in Section 4. Performance evaluations are shown in Section 5. In Section 6, the result and discussion are described. The conclusion is drawn and future enhancement is discussed in Section 7.

## 2. Overview and Architecture

Among the array of many applications that are enabled by the Internet of things (IoT), good and connected health care could be a necessary topic among these applications. The Internet of things (IoT) was initiated in 1959 but the major development in this field was seen in the last 8–10 years. Telemedicine has been used in the treatment of cardiac issues, trauma, and diabetes. Douglas was one of the earlier researchers who determined the importance of telemedicine. His work emphasizes the correct use of resources in an efficient way to improve the health care system. He used the method of store and forward for the transmission of medical information.

The article "Integration of 5G and Block-Chain Technologies in Smart Telemedicine Using IoT" was published in 2021. Journal: J Healthc Eng.

### 2.1. Background

#### 2.1.1. Telemedicine

The use of video conferencing in psychiatry began during the 1950s. In 1950, Norfolk, the Nebraska psychiatric institute, was using early video conferencing to provide group therapy, long-term therapy, consultation-liaison, psychiatry, and medical student training. By the 2000s, outcome studies provided a platform for practice guidelines (e.g. American Telemedicine Association) [2, 3]. APA and ATA have helped to disseminate information on guidelines in the organization. Telemedicine sites are helpful in the progress of telemedicine advancement. Telemedicine sites are listed below:

- American Telemedicine Association (ATA)
- Association of Telemedicine Service Provider (ATSP)
- Telemedicine Information Exchange (TIE)
- NASA Telemedicine
- US DOD Telemedicine
- International Society for Telemedicine (ISFT)
- Telemedicine Association

Figure 2 represents the trend of telemedicine services in recent years. The trend of using telemedicine services is found the most in offices where people with busy schedules can easily contact and narrate their disease symptoms to doctors and get treatment and also be advised on precautions without wasting time waiting for the doctor and also avoid traveling expenses [4]. Telemedicine services are beneficial for the people who are stuck in any extreme weather conditions and cannot go far away for the checkup and treatment; they can visit the nearest health center and get treatment.

In an emergency, telemedicine services help in saving lives specifically in an emergency situation by a timely diagnosis, providing a patient useful information related to his disease and saving the patient's life before a patient faces serious health condition. [5, 6]. The services of Telemedicine are beneficial for the people of rural areas where no hospital, highly equipped laboratories, or medical stores are available [7]. So, in rural areas, during an emergency, people can visit the nearest healthcare center and can get treatment.

#### 2.1.2. Internet of Things (IoT)

Internet of things (IoT) is a wide network that is also implemented in medical devices. IoT devices help in capturing patient's data in a continous manner in a user-centric environment and send data to a cloud platofrm for various health applications whichare used for self-monitoring of patients [8, 9]. This goes hand in hand with the concept of Telehealthcare with devices ranging from wearable to talking devices and wireless monitoring services [10, 11].

The main benefit of IoT is that it is vital to access information and it helps to avoid an emergency. People are more than willing to monitor and control their health at home due to their busy schedules. Internet of things (IoT) devices is meant for remote monitoring in the healthcare sector, to keep the patient safe and healthy, and to empower the medical practitioner to deliver immediate care to the patients [12]. It has increased patient satisfaction as interactions with doctors have become easier and more efficient. Furthermore, remote monitoring of patient's health helps to reduce the visits to the hospital and keep track of patient health records. IoT also has a huge impact on reducing healthcare costs and improving treatment outcomes [13].

The article "Integration of 5G and Block-Chain Technologies in Smart Telemedicine Using IoT" was published in 2021. Journal: J Healthc Eng.

#### 2.1.3. Block-Chain

Block-chain has a wide range of applications and uses in healthcare. The ledger technology facilitates the secure transfer of patient medical record, manages the medicine supply chain, and helps healthcare researchers to unlock the genetic code. Block-chain has a range of built-in features, such as distributed ledger, decentralized storage, authentication, security, and immutability, and has moved beyond hype to practical applications in industry sectors such as healthcare [14]. Block-chain ability to keep an incorruptible, decentralized, and transparent log of all patient data makes it a technology rife for security application. In addition, while block-chain is transparent, it is also private, concealing the identity of any individual with the complex and secure codes that can protect the sensitivity of medical data. The decentralized nature of the technology also allows patients, doctors, and healthcare providers to share the same information quickly and safely [5].

Similarly, text interpreting medical image, with other associated patient information, is included into or acquired directly in digital form and stored. It is important to note that greater the amount of clinical data available to the specialists, acquired, for example, on previously treated cases, better the quality and the rapidity of diagnosis and treatment [15]. It is therefore important, if not essential, to share easily and quickly data and clinical experiences. However, such sharing among different entities, whether public or private, is a nontrivial task, since such information is always subjected to restrictions related to privacy laws and health insurance regulations. To the best of our knowledge, in literature, there are no systems that allow for the rapid and secure sharing of clinical experiences among different entities [15].

Block-chain technology can be very helpful in integrating healthcare information, which is currently scattered, with a range of service providers [16]. Since it is a distributed network, a block-chain-based system can be useful for the integration of several intermediaries in the medical care system. One of its major advantages is interoperability among institutions and service providers. Block-chain can result in improving data integrity, decentralized, and help in delivering precision medicine, improving patient care and outcomes, and connecting medical records across a nation.

The article "Integration of 5G and Block-Chain Technologies in Smart Telemedicine Using IoT" was published in 2021. Journal: J Healthc Eng.

#### 2.1.4. 5G

5G is the fifth generation of cellular wireless technology, which can offer massive connection power and fast Internet speed for data transfer. Patient real-time information is important data for doctors to decide in critical situations. For instance, telemedicine requires an advanced network that offers support in real-time, providing high- quality video communication without slowing down the facility network. Integration of 5G network in existing infrastructure provides real-time data transfer of images, documents, and real-time videos for video-based medical consultations, to improve the quality of care. By using 5G technology, the data transmission rate is high and increases response time that can provide an efficient healthcare system.

Fifth-generation (5G) aims at utilizing many promising communication technologies such as software-defined network and cloud computing technologies. Therefore, secure mechanisms and protocols are required as the basis for 5G networks to address these security challenges and follow security-by-design but also security-by-operations rules [17].

### 2.2. An Architecture of 5G and Block-Chain

In this model, the patient is continuously observed by a lightweight and compact sensor network. In the design of the health care model, the need for security is also considered. An online health care monitoring model ispresented in this paper where sensors collect the patient's data; the patient'shealth data is analysed using machine learning algorithms, and the patient diagnsosis and possible medication details are communicated to a patient in fast and secure manner i [18, 19]. The system works bycollectinga patient's health data, that is needed for the investigation and diagnsosis of a disease. The patient's health datais acquired by sensing and health monitoring devices. The communciation and security aspects of the proposed model is implemented by using 5G services and blockchain technolgies, respectively[20].

 A mobile application isdevloped in Android is used for monitoring a patient's health conditionspecifically in remote areas with the help of a data sensing model for elder people and people with disabilities [4, 21]. The main focus of this model is to give the earliest response in a critical condition of a patient. Figure 3 illustrates the overall architecture of the proposed system. In the first step, the data of the patient are gathered by sensors, medical devices, and can also be obtained by patient history and UCI repository. The gathered data of the patient are stored in a database. The block-chain technology is implemented on data stored in the database, and then data stored in blocks remain secured and help in ensuring privacy with utmost transparency [22, 23]. These secured data are then stored in cloud storage and data in cloud storage are also stored in secured storage so that they would be of help in the future for the treatment of patients by checking their previous data. The data in cloud storage are also forwarded to healthcare providers by using 5G services. The healthcare providers are the end-users who suggest the treatment for the patient. Furthermore, the main purpose of the system is to provide the best time response to the patient for treatment with privacy and secrecy of data.

The article "Integration of 5G and Block-Chain Technologies in Smart Telemedicine Using IoT" was published in 2021. Journal: J Healthc Eng.

The reviewed healthcare applications provide an environment in which billions of users receive information about their health on a daily basis in a periodical manner for a good healthy life [21]. All existing models used various methods for predictions and identification of disease. In this paper, the use of IoT devices and cloud computing in the field of medicine has introduced many features of these applications. In the proposed system architecture, data is collected from different sources such as wearable devices and body sensors that collect data of a patient's health. The other source of patient data is the dataset that is collected through mobile healthcare application. The mobile healthcare application collects the data from body sensors and makes a dataset of body parameter values. The data that are collected from different sources are now stored in the database and the block-chain technology is implemented such that the data become more secure, reliable and interoperable. The secured data of the database is now forwarded to the cloud database server (CDS). The patient data in the cloud database server are stored in a secured storage, which can be of help in future treatment and also show the record of patient history. The data in the cloud database server are analyzed and implemented in the Neural Network algorithm for identification and prediction of result. Neural Network is trained by using atraining dataset, and it is trained enough to predict accurate results. Neural Network predicts results on testing the dataset and identifies that a person is either normal or has a disease condition.

## 3. The Proposed Model

The designed model in this proposed approach is smart and intelligent enough that it's used for prediction and identification of disease and helps in the treatment of disease. Through this system, it's identified that a person's body parameter values are normal or threshold values. Using real-time data of patients, we can identify whether a person has a disease or not. The proposed system is defined by using different sections. Ambient sensor data are collected from different sensors. Different body sensors are used for collecting the body parameter values. The collected data are sent to the cloud server for storage and analysis. Then, an algorithm known as Neural Network analyzes the data and predicts the result as to whether the person is normal or has threshold values of body parameters, which are indicative of the disease. On the server side, the CDSS system is installed in which information on the treatment of diseases are stored. If the symptoms of the disease keyed in match with the data that are stored in the CDSS, then the CDSS will suggest the treatment. If the symptoms of the disease do not match with the data stored in the CDSS, then a query will be forwarded to specialist. The specialist then suggests the treatment. For security purposes, the block-chain technology is used. This makes the system more reliable and secure, and produces robust results. In this proposed system, 5G technology is used. This makes the system faster, efficient, unique, and better compared to all previous systems of healthcare.

The article "Integration of 5G and Block-Chain Technologies in Smart Telemedicine Using IoT" was published in 2021. Journal: J Healthc Eng.

### 3.1. System Architecture

The overall architecture of the proposed model is given (see Figure 3). The main elements in the proposed model are IoT devices, sensor-based application for gathering information, patient medical record, cloud database server (CDS), 5G and block-chain modules, data gathering module, and disease prediction module. The sensor-based application is used and the patient keys in the symptoms of the disease and the body factor parameters that are calculated. The sensors work as a gadget through which the disease of any patient can be predicted. The medical dataset contains the previous record of the patient, which is received by the patient by implementing the block-chain technologies through which data will remain secured and then data are forwarded to healthcare providers by using 5G services.

Dataset disease analysis and previous treatment help in further treatment. These datasets are saved in a cloud database server (CDS). The data gathering module has a vital role in gathering essential data from CDS. The security mechanisms recollect the data from the data gathering module. These data will be saved in a secure manner bypassing various levels of information retrieval, format conversion, and data integration. The secured data saved can be retrieved when required. For flexible access, the essential data are saved in CDS and it helps in disease prediction and treatment. The Disease prediction module used the NN for the prediction of disease. During the training phase, the gathered data from the patient medical record as well as the dataset are used to train the NN classifier.

The article "Integration of 5G and Block-Chain Technologies in Smart Telemedicine Using IoT" was published in 2021. Journal: J Healthc Eng.

During the testing phase, the classifier of the NN specifies the patient data online and predicts after analyzing whether the patient is normal or is affected by any disease. The proposed IoT with a cloud-based CDSS model is based on three levels. In the first level, the required data are gathered from various sources like IoT devices, sensor-based applications, dataset, and patient medical records. They are stored in the database, and the Block-chain technology is implemented, which keeps the data secured. These data are then stored in cloud storage. In the second level, the gathered data that are obtained from different sources are saved in CDS in a secured manner. Then, the data are forwarded to healthcare providers by using 5G services. In the third and final level, the presence of any disease is predicted. It also identifies the level of severity by the use of the NN and previous patient medical records.

### 3.2. Data Gathering

The proposed framework contains three types of data that are gathered from different sources. In this level, the data of different body parameters are gathered by using sensors. When medical sensors are attached, the body parameters are measured and values are calculated. The values are calculated and stored in the database, and the patient data are stored in the database. The block-chain technology is then implemented through which data will remain secured and stored in Cloud storage. The sensor-based values check whether the health care values are normal or not. If body factor parameter values are crossing the normal values, then an alert is raised and calculated values are automatically sent to the doctor for further processing.

The dataset of different body factors calculated will help in further treatment. Another biggest source of data gathering is obtained data of patients from previous records of the hospital. From the previous record of the patient, one can analyze the data and suggest the treatment according to the standard charter of the health plan. The previous record of a patient helps in providing better treatment for the patient. So, in the proposed model, patient data are collected from three different sources, namely, through medical sensors attached to the body, data are gathered from the dataset, and data are gathered from the previous record of the patient.

The article "Integration of 5G and Block-Chain Technologies in Smart Telemedicine Using IoT" was published in 2021. Journal: J Healthc Eng.

Figure 4 is a small module of an overall system architecture that represents the flow graph of how patient body parameter values are calculated by using the sensor-based application. The body parameter values are collected and stored in the database. The block-chain technology is implemented on the patient record that is stored in the database.

Block-chain technology provides transparency and security to healthcare data. The secured data are forwarded to cloud storage where data can be used for frequent treatment and can be stored as patient records, which can be helpful for treatment in the future. The data in cloud storage are forwarded to healthcare providers/experts by using 5G technology. The usage of 5G technology in the proposed system increased the efficiency of the healthcare system.

### 3.3. Sensor-Based Data Collection (Hardware Detail)

The first step for designing this system is to collect information from sensors such as pulse rate sensor, body temperature sensor, oxygen concentration MAX30100 sensor, and blood pressure sensor. The purposed system has a device and also a perception layer that includes hardware devices (sensors, microcontrollers, actuators, and WIFI-devices). The Connectivity layer, application layer, and management layer play a vital role in connectivity, management, and controlling different services in the purposed system. The connectivity layer connects the networking components and manages the network and WIFI modules. The management layer handles the cloud storage by using device management that provides channels for information of data between hardware devices and users (patient, healthcare person) and also cloud through which remote server provides high-level processing [24]. An application layer resides at the top, and it provides features like patient monitoring, checkup scheduling, an indication of body temperature, and notifies the disturbance in body parameters.

Figure 5 represents the processing of sensor data of the system. It contains hardware devices such as sensors, microcontrollers, and smart devices. In Figure 5, on the left side, there are a blood pressure sensor, body temperature sensor, and pulse-rate sensor that are connected with digital input to the microcontroller. The functionality of the microcontroller is like a centralized device that takes inputs from different sensors and data stored in a database, and implements the block-chain technology, which keeps the data secured, and then stores data in the cloud by using the Internet transmit 5G services.

The server processes the data provided by the microcontroller and forwards it to the expert system. The expert system analyzes the data and matches the data with stored data. Probably, treatments can be suggested in three ways according to the case on hand. First, if an expert system has information about the disease, the symptoms of which are received, then the expert system suggests the treatment. Second, otherwise, data are forwarded to the specialist who then recommends the treatment for the patient within 24 hours. Third, if the patient has a disease, the symptoms of which are not stored in the expert system and the specialist also has no information about the disease, then the specialist consults with a panel of doctors. The panel of doctors hold meetings and exchange information about the disease, make experiments, and collect all possible information relevant to the disease, and after the conclusion, treatment is recommended to patients through the healthcare center or by the expert system via the Internet. The expert system is updated by storing information and treatments about new diseases.

The article "Integration of 5G and Block-Chain Technologies in Smart Telemedicine Using IoT" was published in 2021. Journal: J Healthc Eng.

#### 3.3.1. Arduino Uno Microcontroller

We used an open-source microcontroller board (as shown in Figure 6) composed of 14 digital and 6 analog input/output (I/O) pins, which can be used to communicate various expansion boards (shields). These pins can be programmed with the Arduino IDE (Integrated Development Environment) by using a type B USB cable.

The following are key features of the Arduino UNO Microcontroller:

- 6 analog inputs
- Operating Voltage: 5 V
- Input Voltage (Recommended): 7–12 V
- Input Voltage (Limit): 6–20 V
- DC current for 3.3 V pins: 50 mA
- Microcontroller: AT mega328

#### 3.3.2. Pulse-Rate Sensor

The pulse rate is used to detect and calculate the pulse rate of a human being. Experts recommend this sensor for real-time monitoring of the heart rate. It's also called a biometric pulse rate or heart-rate detecting sensor. The pulse-rate sensor is used for anxiety monitoring, health bands, sleep tracking, advanced gaming consoles, and remote patient monitoring/alarm system. A typical pulse-rate sensor is shown in Figure 7.

The following are key features of a pulse-rate sensor used in monitoring the pulse rate of a human being.

- Operating voltage: +5 V or +3.3 V
- Current consumption: 4 mA
- Diameter: 0.625″
- Thickness: 0.125″ thick
- Inbuilt amplification and noise cancellation circuit
- Biometric pulse rate or heart-rate detecting sensor
- Plug and play type sensor

#### 3.3.3. Blood Pressure Sensor

The blood pressure sensor is used to calculate the pressure in veins. A blood pressure sensor provides accurate values of blood pressure. A typical blood pressure sensor is shown in Figure 8.

The article "Integration of 5G and Block-Chain Technologies in Smart Telemedicine Using IoT" was published in 2021. Journal: J Healthc Eng.

The following are key features of a blood-pressure sensor

- Plug and play type sensor
- Normal values lie between 80 and 120
- Provides information about blood rate
- Blood rate detecting sensor

#### 3.3.4. The MAX30205 Body Temperature Sensor

The MAX30205 is used to measure human body temperature. The MAX30205 body temperature sensor is a digital thermometer that is accurate to measure body temperature. The resolution of MAX30205 is 16 bits (0.00390625°C), as shown in Figure 9.

The following are key features of the human body temperature sensor MAX30205

- 0.1°C accuracy
- Operating supply current (600 A)
- Voltage range from 2.7 V to 3.3 V
- Temperature resolution: 16-Bits
- Operating temperature range: 0°C to +50°C
- One-shot, shut down modes for reduced power consumption
- A selectable timeout prevents bus lockup
- 8-pin TDFN package (0.65 mm pitch)

#### 3.3.5. Oximeter MAX30100 Sensor

The MAX30100 is a Pulse Oximeter sensor (see Figure 10) that measures oxygen saturation level in the body. Oxygen is used to breathe and there is also a need for oxygen in the body. Because of the deficiency of oxygen in the body, cells of the body will deteriorate, organ failure will occur, and ultimately death occurs. The purpose of the Max30100 pulse oximeter sensor is to measure the oxygen found in hemoglobin, protein. The normal oxygen saturation level lies between 95 and 100%.

The following are key features of the MAX30100 pulse Oximeter sensor

- Efficient, painless, and noninvasive
- Able to notify the patient of oncoming and existing low oxygen saturation level in the blood
- Records oxygen saturation trends (physical activity) of the patient and can adjust the oxygen level where necessary
- Effective in keeping oxygen use accurate
- Essential in monitoring illnesses

### 3.4. Integration of 5G with Block-Chain Technologies

With the progress in electronic health-related data, cloud healthcare data storage, and patient data privacy protection regulations, new opportunities are opening for health data management, with regard to patients' convenience to access and share their health data. Three important qualities of block-chain are:

- Decentralization
- Immutability
- Security

One area that could greatly benefit from block-chain technology is Telemedicine, the relative field of providing remote delivery of healthcare services over telecommunication [15]. Block-chain technology allows healthcare professionals to access the desired information in a decentralized ledger. This integration of 5G and block-chain technologies also allows for the elimination of information blocking. Ideally, this would provide patients the ability to access their medical records when needed and to securely share the information with their doctors.

The article "Integration of 5G and Block-Chain Technologies in Smart Telemedicine Using IoT" was published in 2021. Journal: J Healthc Eng.

There have been security concerns when it comes to telemedicine. If the connection between the doctor and patient is not secure, it increases the risk of data breach [14]. Block-chain and 5G technologies when applied in the given scenario create a secured network. Block-chain technology also stores the medical record in a secure, fragmented system that contains a large amount of data and information, enabling providers to store more completed patient history and securely encrypted medical records. The architecture is shown in Figure 11.

Deployment of 5G will bring in great benefits like faster data transmission, seamless data loaded files download capability, remote monitoring of smart devices, and real-time telemedicine visits. The 5G initiative improves all hospital processes and breaks the main barrier of Internet bandwidth, creating truly smart hospitals. Furthermore, the deployment of 5G with block-chain technologies will allow medical staff to exchange information with patients securely and at a fast transmission rate.

Figure 11 illustrates the integration of 5G and block-chain technologies in the Telemedicine healthcare system.

- Step-1: in this proposed system, the patient is a source of data. Patient data are collected using sensors or medical devices. The correct measurement of patient data is a necessary parameter of this proposed system.
- Step-2: sensors or medical IoT devices are normally attached either closely or remotely to monitor patients' body, consequently, generating a large volume of data. Analyzing the patient data helps to provide better treatment.
- Step-3: data gathered in step-2 are stored at a storage point that can be a database of patient data and then data can be stored in blocks by securely using block-chain technology for data security. The secured data of the patient is stored in the cloud for future purposes and helps in providing better treatment by checking the previous record of the patient. The data are forwarded with the highest transmission rate to healthcare providers by using 5G services. A result of high transmission rate of data has the highest response time that is effective in the healthcare system. In the case of sensitive data where security is the priority, a secured database with centralized block-chain technology helps to have the highest security.
- Step-4: healthcare providers are the end-users who seek access to safe and sound care delivery. Healthcare providers play a vital role in providing healthcare services to patients according to their disease.

### 3.5. Security Mechanism on CDS

The proposed framework contained three types of data that help in decision-making. The three types of data contained the data that are obtained from the IoT-based sensor application. Dataset and the patient record were obtained from the hospital based on the severity level of disease. These three kinds of data have been stored in the database and used for further process and investigation. The cloud platform gives enough space to store a large amount of data [25].

The article "Integration of 5G and Block-Chain Technologies in Smart Telemedicine Using IoT" was published in 2021. Journal: J Healthc Eng.

The proposed security mechanism intends to secure healthcare data efficiency [25]. In the healthcare system, the security mechanism is a necessary component. For security mechanisms, block-chain technology is used to secure the data of patient health records. The block-chain is one such technology that can maintain an incorruptible ledger to store health records and allow patients and healthcare institutes to manage information transparently [17].

In the proposed system, security mechanism on Clinical Decision Support is provided by block-chain technology. Block-chain technology is applied to patient records stored in the database, and data are fragmented into different blocks so as to ensure the transparency of data. Secured data are stored in cloud storage and forwarded to healthcare providers by using high transmission of 5G technology.

#### 3.5.1. Clinical Decision Support System

A clinical decision support system (CDSS) is an application that analyzes the data and provides help to healthcare personnel to make a decision and provide support in improving the health of a patient [26]. Clinical decision support systems enable integrated workflows to provide care plan recommendations and assist at the time of providing care.

The focus of the CDSS on using knowledge management for getting clinical advice is based on multiple factors of patient-related data. When using a clinical support system, data mining can be conducted to analyze whether the medical history of a patient is in conjunction with data relevant to the clinical research.

A traditional CDDS comprises software designed to be a direct aid in clinical decision-making, in which the characteristics of an individual patient are matched to a computerized clinical knowledge base, and patient-specific assessment or recommendations are then presented to a clinician for a decision.

In this proposed system, the clinical decision support system (CDSS) plays a vital role in the healthcare system. The experts store the treatments of many diseases in the CDSS. If the symptoms of the patient disease match with the record of the CDSS, then the CDSS suggests the treatment for the relevant disease. If patient disease symptoms are not matched with the record that is stored in the CDSS, then the CDSS forwards the patient data to healthcare providers for suggestions/treatment of the disease.

The article "Integration of 5G and Block-Chain Technologies in Smart Telemedicine Using IoT" was published in 2021. Journal: J Healthc Eng.

#### 3.5.2. Components of the CDSS

A typical CDSS comprises three vital components, as shown in Figure 12:

1. Data repository
2. Rules engine
3. User interface

*(1) Data Repository*. The data repository holds all data and information contents required by the CDSS and the CDSS forwards meaningful information to users related to the disease. The content can be in three forms: structured knowledge data, structured or unstructured data in text material, or content could be processed structured data from EPR application themselves.

*(2) Rules Engine*. Rules engine is helpful in analyzing and interpreting the knowledge as it is a central component of the CDSS. The rules engine is capable of analyzing patient data, but files of patient data are not stored in the rules engine. During the process, the clinical rules engine activates and interprets the relevant protocol. .

The rules engine understand the content, like

- Medication dosage in relation to kidney functioning
- In the case of heart medication, electrolytes used
- In the case of cardiac arrest, the choice of anti-coagulate is available

*(3) Interface*. User interface is a sophisticated part of the clinical decision support system (CDSS) and also plays a vital role in establishing communication between sensor-based application and the CDSS. The interface can be of two types:

- User-interface collects real data that is stored in a repository and analyzed bya rule engine and then commnicated to a user.
- *Service-based* A service-based interface of the CDSS provides data ideally as XML back to the sensor-based application for it to process the output on its own.

#### 3.5.3. Architecture of the CDSS

The architecture of a clinical decision support system consists of the following ten components:

- Knowledge authority environment
- Electronic medical database
- Case database
- Machine learning
- Inference engine
- Query engine
- User interface
- Knowledge base
- User
- Patient data

The architecture of the used CDSS is shown in Figure 13:

#### 3.5.4. Efficiency of the Proposed Model over the Existing Model

The proposed model is more efficient in working, response, and security than the existing model. In the proposed model, the time factor is minimized by using the modern technology in which the patient can calculate the body parameter values by using a sensor-based application and can forward the data to an expert system or physician. One more efficiency of the proposed model than the existing model is the usage of an expert system like the CDSS. Many treatments can be suggested through the CDSS system, and for the treatments that are not present in the CDSS, the CDSS forwards the data to an expert/specialist for treatment.

The article "Integration of 5G and Block-Chain Technologies in Smart Telemedicine Using IoT" was published in 2021. Journal: J Healthc Eng.

*Comparison*
  - In the existing model, the patient needs to visit the nearest healthcare center where the healthcare person conducts a checkup on the patient and calculates the body parameter values of the patient, and forwards the data to the doctor/physician through e-mail. The patient needs to visit the healthcare center 2–3 times and then the healthcare person suggests the treatment according to experts' suggestions. But, the existing system is not efficient because it's expensive and takes more time for treatment. The existing model is not efficient because it's expensive as a clinic/healthcare center and staff for healthcare centers must be present in rural areas. The existing model is also not efficient for a patient because it involves more time and money.
  - The proposed model is better than the existing model because healthcare centers or healthcare personnel are replaced with the smart IoT sensor-based mobile application. Now patients, without going to healthcare centers, can send data through the mobile application. A patient can touch the sensor-based application or manually enter the body parameters data and forward it to the specialist; then, the specialist suggests treatment according to the disease.

## 4. Neural Network and Prediction System

In this section, the proposed neural network predicts the disease and determines the severity level. The proposed model decides on healthcare data. The benefit of this proposed model is the selection of attributes and classification of medical records depending upon the time limitations for making decisions effectively.

An Artificial Neural Network (ANN) is a computationally intelligent technique that is stimulated from the network of biological neurons for natural language processing, for prediction of problem-solving, identification of severity level, and so on. In our proposed approach, we used the neural network for classifying the current environment for efficient prediction of disease [27]. Although there are many machine learning algorithms, e.g., SVM, Random forest, decision tree, KNN, etc., which could provide solutions for classification problems, we preferred the neural network to other machine learning approaches due to many reasons.

- The first reason is that the NN (Neural network) can handle a large amount of training dataset, as in this scenario the number of cases and experimental sets may increase in the future.
- The second reason for preferring the neural network to other machine algorithms is flexibility as new features can be added by increasing data size, which ultimately reflects in the output.
- The third reason for choosing the neural network (NN) is its ability to outperform other machine learning techniques.
- The fourth reason for the preference of neural networks is that the NN is suitable for nonlinear problems, as the current problem cannot be solved by a separable linear function.

The article "Integration of 5G and Block-Chain Technologies in Smart Telemedicine Using IoT" was published in 2021. Journal: J Healthc Eng.

An Artificial Neural Network is a famous technique of machine learning that was first developed in 1950 [28]. An ANN provides high accuracy results of prediction. They have capabilities of efficient decision-making like a human which is why it's best suited in medical decisions like prediction and pattern recognition. The most famous application of neural networks in the medical domain is clinical diagnosis, image analysis, and interpretation. A Neural Network (NN) addresses the problem of supervised learning, i.e., a dataset contains all possible examples of input data with their accurate truth values, and the output is provided. A Neural Network (NN) learns this dataset pattern and could be used to predict class/labels of incoming dataset where class/labels are not known. Furthermore, the NN provides a classification layer above stored data. A neural network consists of three components.

- Input layer
- Hidden layer
- Output layer

There are many types of neural networks (NN) to use, i.e., conventional neural network, backpropagation, feedforward, etc. Learning of the NN consists of forwarding propagation and backpropagation.

The configuration of the NN takes place by modifying the following parameters: the number of hidden layers, the activation function, and the number of learning steps [29]. For every manual configuration, the validation of classification accuracy takes place over the testing set. The NN classifier class employed here generates all neuron layers, using the ReLU (Rectified Linear unit) activation function. From equation (1) function, it's seen that the NN is simpler and effective, as shown in Figure 14.

The output layer depends upon the Softmax function, and the cost function is cross-entropy. The rectifier is an activation function represented in equation (1).

(1) $$\begin{array}{c} f\left(x\right)=x+=\max\left(0,1\right), \end{array}$$

where *x* is the input of neurons. It is also called a ramp function, which is similar to the half-wave rectification process in electrical engineering. A unit utilizing the rectifier is termed as the Rectified Linear Unit (ReLU). A smooth approximation of rectification is an analytical function:

(2) $$\begin{array}{c} f\left(x\right)=\ln\left[1+\exp\left(x\right)\right], \end{array}$$

which is called soft plus function. The rectifier and soft plus function are illustrated in Figure 15. During the prediction process, a new representation of raw descriptors is filtered from hidden layers as follows:

(3) $$\begin{array}{c} X_{t+1}=H\left(W_{l}X_{l}+B_{l}\right),\;l=1,\ldots ,1, \end{array}$$

where *W*_*l*_ and *B*_*l*_ represent the weight matrix and bias of the hidden *l*th layer, and *H* is the related activation function, which is chosen to be the rectified linear unit (ReLU). Figure 15 shows the plot:

The pseudo-code explaining the steps in the NN (Neural network) classifier is given below.

- Load the training and testing dataset.
- Construct the NN classifier utilizing chosen for manual configuration, i.e., activation function, number of learning steps.
- Estimate the accuracy of the NN in the testing set.
- Compute the prediction of the NN.
- Assess the classification results of the NN in the testing set using the confusion matrix
- Validate the classification result of the NN on the entire dataset.

The article "Integration of 5G and Block-Chain Technologies in Smart Telemedicine Using IoT" was published in 2021. Journal: J Healthc Eng.

## 5. Performance Evaluation

For assessing the classification result of the NN classifier on a dataset, a set of experiment datasets are carried out. The proposed model has been implemented by using the python program. The detail of datasets, performance evaluation, and results are discussed in the following subsection.

### 5.1. Dataset Details

The proposed model is validated by employing the dataset obtained from various sources. The detail of the dataset is tabulated in Table 1.

The dataset holds a total of 700 instances, 4 attributes, and two classes, namely, continuous and impaired. From the total of 700 instances, 470 instances came under the continuous class and the remaining 230 came under the impaired class. In this case, 470 instances are employed for testing, and 230 instances are employed for testing purposes. The purposed model is trained for the testing of the dataset. This procedure splitting the dataset for training and testing will be reiterated for up to ten minutes.  Table 2 shows the dataset instances for which the system is trained.  Table 3 shows the training dataset.

Table 4 shows the dataset detail that is used for training the Neural Network. The Neural Network is trained by defining the different rules. Some of the rules are defined below:

- IF (Blood Pressure = = Very High) AND (Pulse Rate = = Normal) AND (Temperature = = Very High) AND (Oxygen Concentration = = High) ,THEN Decision = High
- IF (Pulse Rate = = Normal) AND (Temperature = = Normal) AND (Blood Pressure = = Medium) AND (Oxygen Concentration = = Normal), THEN Decision = Low
- IF (Temperature = = Normal) AND (Pulse Rate = = Normal) AND (Blood Pressure = = normal) AND (Oxygen Concentration = = High), THEN Decision = Low
- IF (Temperature = = Normal) AND (Pulse Rate = = High) AND (Blood Pressure = = High) AND (Oxygen Concentration = = High), THEN Decision = High
- IF (Pulse Rate = = High) AND (Temperature = = Normal) AND (Blood Pressure = = Low) AND (Oxygen Concentration = = Low), THEN Decision = Low

The article "Integration of 5G and Block-Chain Technologies in Smart Telemedicine Using IoT" was published in 2021. Journal: J Healthc Eng.

#### 5.1.1. Designing the Neural Network

To train the neural network, the training data-set is implemented by employing the following steps:

(i) Import the training dataset
(ii) Import the target dataset
(iii) Do necessary configuration of the network
  1. Input layer
  2. Hidden layer
  3. Activation function
(iv) Start training
(v) Repeat training to gain maximum performance
(vi) Export model
(vii) Check performance

First of all, import the trained dataset, the training dataset that trained the NN (Neural Network). This NN tool required the input dataset and target dataset for training. We import both input and test data variables into the workspace. And, then we add a Neural Network and set properties as required by the design that is discussed in Section 3. A chunk of the dataset is shown in Figure 16.

### 5.2. Measures

For highlighting the classification result of the proposed model using the NNN classifier, a set of performance measures used includes the false-positive rate (FPR), false-negative rate (FNR), the area under the curve (AUC), specificity, *F*-score, Mathew correlation coefficient (MCC), and kappa value. Before defining the measure of classification, define the confused matrix. A confused matrix is defined as a 2 ∗ 2 matrix, comprising 4 elements, namely, true positive denoted by TP, true negative denoted by TN, false-positive denoted by FP, and false-negative denoted by FN. Classification measures are defined based on the confusion matrix.

FPR is used to compute the possibility of wrongly rejecting the null hypothesis for a specific test. It is represented in

(4) $$\begin{array}{c} \text{FPR}=\frac{\text{FP}}{\text{FP}+\text{TN}}. \end{array}$$

FNR is used to compute the conditional probability of a positive test result given an instance that was not present. It is the ratio of the total number of correctly classified instances, and the false instances are classified as negative. It is represented in

(5) $$\begin{array}{c} \text{FNR}=\frac{\text{FN}}{\text{FN}+\text{TN}}. \end{array}$$

The sensitivity indicates the number of actual positives that are correctly classified as positive and is represented in

(6) $$\begin{array}{c} \text{sensitivity}=\frac{\text{TN}}{\text{TN}-\text{FP}}. \end{array}$$

Specifically represent the number of actual negatives, which are correctly classified as negative and are represented in equation (7)

(7) $$\begin{array}{c} \text{Specificity}=\frac{\text{TN}}{\text{TN}+\text{FP}}. \end{array}$$

Accuracy is the most widely used classification performance metric. It represented the number of instances that are positive and show the percentage of these instances. For better classification performance, the classification accuracy should be closer to 100% and is defined as represented in

(8) $$\begin{array}{c} \text{accuracy}=\frac{\text{TP}+\text{TN}}{\text{TP}+\text{TN}+\text{FP}+\text{FN}}. \end{array}$$

*F*-score determines the accuracy of the testing process. It is an average measure and is used for decision and recall for the dataset, as shown in

(9) $$\begin{array}{c} F-\text{score}=\frac{2\text{TP}}{2\text{TP}+\text{FP}+\text{TN}}. \end{array}$$

MCC is a balanced metric typically used when the classes have various sizes as given in equation (10).

(10) $$\begin{array}{c} \text{MCC}=\frac{\left(\text{TP}.\text{TMN}-\text{FP}.\text{FN}\right)}{\;\sqrt{\left(\text{TP}+\text{FP}\right)}\left(\text{TP}+\text{FN}\right)\left(\text{TP}+\text{FP}\right)\left(\text{TN}+\text{FN}\right)}. \end{array}$$

Kappa coefficient value (*K*). Kappa computes the value of agreement between two classifications in which it classifies N item into C mutually exclusive categories.

(11) $$\begin{array}{c} \text{Kappa test}=\frac{\text{observed agreement}-\text{expected agreement}}{100-\text{expected agreement}}, \end{array}$$

where observed agreement = % (overall accuracy)

(12) $$\begin{array}{c} \text{expected agreement}=\left(\%\left(\text{TP}+\text{FP}\right)*\%\left(\text{TP}+\text{FN}\right)\right)+\left(\%\left(\text{FN}+\text{TN}\right)*\%\left(\text{FP}+\text{TN}\right)\right). \end{array}$$

The comparison of the classification results in terms of FPR and FNR are shown in Figure 17, where it is depicted that the values for MLP is higher for both FPR and FNR. Similarly, Figure 18 shows the comparison of the classifier result in terms of various measures.

The article "Integration of 5G and Block-Chain Technologies in Smart Telemedicine Using IoT" was published in 2021. Journal: J Healthc Eng.

## 6. Results and Discussion

### 6.1. Performance Evaluation Using the NN with Various Classifiers

Table 5 provides the experimental result proposed NN classifier, multilayer perceptron (MLP), the fuzzy-based neural classifier, and decision tree (DT) in terms of different measures of FPR and FNR, sensitivity, specificity, accuracy, *F*-score, MCC, kappa, and AUC shows the values and result of the NN classifier and other classifiers in terms of FPR and FNR. To attain better classifier results, the value of FPR and FNR should be as low as possible. From Table 5, it is evaluated that among the compared methods, the highest FPR and FNR value is, respectively, 11.25 and 10.39, which is attained by the MLP classifier. These values imply that the MLP classifier has the worst performance. Next, the FNC manages to perform better than MLP and DT classifiers except for those of the NN classifier. Furthermore, the NN classifier attains the lowest value of FPR and FNR of 0.55 and 2.1, respectively.

Table 5 shows the obtained experimental results of different classifiers in terms of six measures, namely, accuracy, *F*-score, AUC, sensitivity, specificity, and Kappa values. For all of these measures, the value should be as high as possible, i.e., closer to 100. The classifier that has the highest value is considered as the best classification algorithm.

In terms of sensitivity, Table 5 shows that the MLP classifier shows a poor result with the lowest value of 90.38, whereas the DT attains the value 92.20. Moreover, FNC tries to achieve maximum performance with a sensitivity value of 94.68. However, it should be only an inferior result to the proposed NN classifier. From sensitivity values, it's concluded that the NN classifier is better than all other compared methods.

On measuring the result of classifiers in terms of specificity, the order of performance of the classifiers is as follows: NN, FNC, DT, and MLP. The MLP classifier lies at the end of the order because the performance of the MLP is poor. The NN classifier lies in the first position of the order because the NN classifier attains a maximum value of specificity.

In Figure 19, the measuring values of sensitivity in terms of different classifiers are shown. The classifier that attains the maximum value of sensitivity has the best performance. According to results, it's concluded that the NN attains the maximum values of sensitivity and specificity compared to all other classifiers. So, the NN shows better performance than all other classifiers.

The accuracy classification classifier is an important metric. The NN classifier obtains a maximum accuracy of 98.98, whereas the MLP classifier attains the minimum value of accuracy 89.11. Similarly, the lowest *F*-score attained by the MLP indicates the worst classification performance with a value of 89.45, whereas FNC and DT showed competitive performance with the *F*-score values of 94.98 and 94.01, respectively. Interestingly, the NN classifier attains an *F*-score value that is higher than all other compared methods. Likewise, the NN classifier attains the highest value in AUC while other methods cannot attain such a high value.

The Kappa value of classifiers (see Figure 20) shows that the MLP fails to show superior results while the NN classifier shows excellent performance than all other compared classifiers. From all results, it's concluded that the NN is a superior classifier than the FNC, DT, and MLP classifiers.

The article "Integration of 5G and Block-Chain Technologies in Smart Telemedicine Using IoT" was published in 2021. Journal: J Healthc Eng.

## 7. Conclusion and Future Work

This paper has presented an IoT with a cloud-based CDSS framework, which was implemented for the prediction of disease and its severity level. Furthermore, medical sensors are utilized for gathering patient data and the previous record of a patient that helps in better treatment of the patient. The gathered data from different sources are stored in the database and then the block-chain technology is implemented, which keeps the data secured and then data are stored in cloud storage. The data securely stored in cloud storage are forwarded to healthcare providers by using 5G services. We used an exterior environment monitoring system to record current environment readings using the Arduino UNO, Max30100 oximeter, blood pressure sensor, pulse-rate sensor, and human body temperature sensor. The next component of the presented model used the NN-trained model, which takes a designed standard training dataset to train the NN to predict the environmental feasibility of data and the result of the class that is not labeled. In the proposed model, the telemedicine system is more efficient than all previous systems, as in this system the critical factors that are influencing the efficiency of the system are controlled. The accuracy of the system is compared with different classifiers and shows that the Neural Network (NN) gives better performance and accuracy than all other classifiers. The proposed approach has many advantages in healthcare services, and few of them are listed below:

- The purposed system is efficient in providing healthcare services more effectively.
- In this proposed system, time is minimized by overcoming the critical factors of the environment.
- The system is also best suited for the people of rural areas where no proper health facilities are provided.
- In this designed system, the potential of block-chain is to overcome the challenges related to data security, privacy, sharing, and storage. Furthermore, block-chain technology in the proposed system ensures that medical data are secured in the healthcare system with the utmost transparency.
- In the given proposed system, usage of 5G services increases the efficiency of healthcare services.
- The system is also best suited for disabled persons, who are not able to travel long distances.

There are many future perspectives enhanced in the proposed healthcare approach, and few of them are mentioned here:

- The proposed approach could be implemented with other algorithms, e.g., KNN. Fuzzy system, and Deep Neural Network.
- In the future, the selection algorithm could be used for optimization and effective results.
- the proposed approach could enhance to cover large patient range by adding their profile.
- In the future, using the PSO (Particle Swarm Optimization) technique as the feature selection will increase the optimization of the system and present the system in a more efficient way.

The article "Integration of 5G and Block-Chain Technologies in Smart Telemedicine Using IoT" was published in 2021. Journal: J Healthc Eng.

## Figures and Tables

**Figure 1:** Store and forward method of telemedicine.

**Figure 2:** The trend of Telemedicine Services.

**Figure 3:** System architecture.

**Figure 4:** Sensor-based data from humans.

**Figure 5:** Processing of sensor data.

**Figure 6:** Arduino UNO microcontroller.

**Figure 7:** Pulse rate sensor.

**Figure 8:** **:** Blood-pressure sensor.

**Figure 9:** Body temperature sensor.

**Figure 10:** MAX 30100 oximeter sensor.

**Figure 11:** Block-chain and 5G technologies in healthcare.

**Figure 12:** Components of the CDSS

**Figure 13:** Architecture of the CDSS

**Figure 14:** Neural network architecture.

**Figure 15:** Plot of the rectifier near *x*, *y* = 0.

**Figure 16:** Import the training dataset.

**Figure 17:** Comparison of classification results in terms of FPR and FNR.

**Figure 18:** Comparison of the classifier result in terms of various measures.

**Figure 19:** Comparative sensitivity and specificity of the NN with other classifiers.

**Figure 20:** Comparative accuracy of the NN with other Classifiers.

**Table 1:** Dataset description.

Detail	Value
Source	Sensors, UCI
# of instance	700
# of attribute	4
# of classes	2
Continues/impaired	470/230

**Table 2:** Data of instances.

Parameters	Instances	Classes
Children 200	150	Continuous
	50	Impaired
Adults 200	140	Continuous
	60	Impaired
Teenage 120	60	Continuous
	60	Impaired
Old aged 180	120	Continuous
	60	Impaired

**Table 3:** Classification of used training data.

Instance	Pulse rate		Body temperature		Oxygen concentration		Blood pressure	
Children 200	Low	20	Low	10	Low	50	Low	40
	Normal	175	Normal	140	Normal	120	Normal	150
	High	5	High	50	High	30	High	10
Adults 200	Low	30	Low	10	Low	50	Low	20
	Normal	120	Normal	160	Normal	50	Normal	170
	High	50	High	30	High	100	High	10
Teenage 120	Low	40	Low	10	Low	30	Low	50
	Normal	50	Normal	90	Normal	70	Normal	20
	High	30	High	20	High	20	High	50
Old aged 180	Low	10	Low	20	Low	60	Low	10
	Normal	100	Normal	80	Normal	50	Normal	70
	High	70	High	80	High	70	High	100

**Table 4:** Training dataset.

SR#	ID	Body temperature (°C)	Pulse rate (BPM)	Blood pressure (mmgh)	Oxygen concentration (%)	Label
1	Gender1	97	61	122/80	92	Normal
2	Gender2	97.5	66	123/83	93	Normal
3	Gender3	98	70	125/82	95	Healthy
4	Gender4	98.3	71	127/82	94	Healthy
5	Gender5	104	72	130/90	96	Threatening
6	Gender6	102	75	129/92	99	Threatening
7	Gender7	102.3	80	134/91	98	Dangerous
8	Gender8	101	76	135/93	97	Threating
9	Gender9	100	74	137/95	92	Threatening
10	Gender10	97.9	73	136/92	93	Threatening
11	Gender11	98.8	81	133/91	100	Dangerous
12	Gender12	97.4	89	140/95	95	Dangerous
13	Gender13	99	83	145/96	93	Dangerous
14	Gender14	102	85	122/85	91	Threatening
15	Gender15	103.4	82	135/91	99	Dangerous
16	Gender16	103.8	76	121/96	98	Threatening
17	Gender17	103.7	79	141/98	97	Dangerous
18	Gender18	98.3	78	145/92	96	Threatening
19	Gender19	102	85	137/85	99	Dangerous
20	Gender20	98	74	123/89	92	Healthy
21	Gender21	101.3	73	122/87	93	Healthy
22	Gender22	101	71	125/80	93	Normal

The article "Integration of 5G and Block-Chain Technologies in Smart Telemedicine Using IoT" was published in 2021. Journal: J Healthc Eng.

**Table 5:** Comparison of classifier results in terms of various measures.

Classifier	FPR	FNR	Sensitivity	Specificity	Accuracy	*F*-score	AUC	MCC	Kappa
NN	0.55	2.1	98.50	99.50	98.98	98.78	98.78	0.98	97.10
FNC	4.01	4.10	94.68	95.87	92.50	94.98	95.90	0.81	90.25
DT	7.10	7.50	92.20	91.45	82.30	94.01	91.45	0.78	81.67
MLP	11.25	10.39	90.38	89.11	79.45	90.0	89.45	6.56	78.21

## Data Availability

The datasets used in the experiments and discussed in the paper are available upon request to the corresponding author.
